The article "Investigation of Interaction between Vitamin D Receptor Gene Polymorphisms and Environmental Factors in Early Childhood Caries in Chinese Children" was published in 2019. Journal: Biomed Res Int.

# Investigation of Interaction between Vitamin D Receptor Gene Polymorphisms and Environmental Factors in Early Childhood Caries in Chinese Children

**DOI:** 10.1155/2019/4315839

**Published:** 2019-12-17

**Authors:** Xiurong Qin, Linqin Shao, Lixia Zhang, Long Ma, Shijiang Xiong

**Affiliations:** ^1^Department of VIP Center, School and Hospital of Stomatology, Shandong University, Shandong Provincial Key Laboratory of Oral Tissue Regeneration & Shandong Engineering Laboratory for Dental Materials and Oral Tissue Regeneration, Jinan, Shandong Province, China; ^2^Department of Pediatric Dentistry, Jinan Stomatological Hospital, Jinan 250001, Shandong Province, China

## Abstract

**Background:**

Early childhood caries is a multifactorial disease involving interactions between genetic and environmental risk factors. The aim of this study was to examine the effects of vitamin D receptor (VDR) gene polymorphisms and gene-environment interactions on the etiology of, and susceptibility to, caries in Chinese children aged 3–5 years.

**Methods:**

Children (*n* = 549) were divided into three groups according to caries risk: high (decayed, missing, filled teeth (dmft) index > 4; *n* = 148), moderate (dmft = 1–4; *n* = 156), and caries-free (*n* = 245). A questionnaire was designed to collect demographic information, dietary habits, and oral hygiene practices, and dental plaque samples were collected to test acidogenic activity of bacteria. Genomic DNA was extracted from the buccal mucosa, and the VDR polymorphisms rs7975232, rs1544410, rs11568820, rs10735810, and rs731236 were genotyped using TaqMan assays.

**Results:**

There were no differences among the caries risk groups in frequencies of the rs7975232, rs731236, rs1544410, or rs11568820 polymorphisms (*χ*^2^ test, *P* > 0.05); however, the frequency of the rs10735810 CC genotype was clearly higher in the high caries risk group than in the control and moderate caries risk groups (39.2%, 25.6%, and 30.6%, respectively; *χ*^2^ test, *P*=0.028). In multivariate analysis of genotypes and behavioral factors, rs7975232, rs731236, rs1544410, rs11568820, and rs10735810 were not associated with deciduous tooth decay (*χ*^2^ test, *P* > 0.05).

**Conclusion:**

We conclude that these VDR polymorphisms cannot be used as markers for identification of Chinese children at increased risk of dental caries, when combined with environmental factors. Future studies are needed to replicate these initial findings and better assess the risk of caries in deciduous teeth.

## 1. Introduction

Globally, early childhood caries (ECC) is the most common childhood oral health problem [1], and the most prevalent childhood disease, occurring five times more frequently than asthma, which ranks second in incidence [2]. In China, the prevalence rates of ECC are 50.8%, 63.6%, and 71.9% in 3-, 4- and 5-year olds, respectively [3]. Untreated ECC can cause serious health problems, including local pain, infections, abscesses, loss of teeth, and malocclusion, leading to speech difficulties, and can seriously impact the psychological and physical health of children [4–6]; hence, ECC represents a major public health problem that urgently requires resolution.

The article "Investigation of Interaction between Vitamin D Receptor Gene Polymorphisms and Environmental Factors in Early Childhood Caries in Chinese Children" was published in 2019. Journal: Biomed Res Int.

ECC is a chronic, transmissible, infectious disease with a complex and multifactorial etiology. Environmental factors, such as cariogenic bacteria, cariogenic diet with a high carbohydrate content, insufficient fluoride exposure, inappropriate methods of infant feeding, poor oral hygiene in children, nutrition, maternal education level, and poverty, have been studied extensively [7, 8]; however, when exposed to the same levels of environmental risk factors, some patients are more susceptible or resistant to caries than others [9, 10], indicating that environmental factors alone are insufficient to explain the condition. Heredity may be another factor linked with caries susceptibility. Although the importance of genetic factors is recognized, to date, only a few caries susceptibility genes have been reported, including factors involved in enamel formation, immune responses, saliva, and taste, among others [11].

Vitamin D (Vit D) plays an important role in enamel mineralization [12], and Vit D supplementation can reduce the risk of dental caries by 47% [13]. The vitamin D receptor gene, VDR, which maps to human chromosome 12q13.1, mediates the effects of Vit D, including maintenance of the calcium and phosphate balance and regulation of mineralized tissue development [14–16]. The VDR gene contains more than 200 polymorphic sites, among which five single nucleotide polymorphisms related to dental caries have been studied: rs1544410, rs731236, rs7975232, rs10735810, and rs11568820 [17–20]. The majority of these studies reported associations between VDR polymorphisms and susceptibility to permanent tooth caries [17, 18, 21]. Based on these literatures, although we can conclude that VDR has a role in susceptibility to dental caries, associations between VDR gene polymorphisms and susceptibility to dental caries vary greatly in different geographical regions, among people of different ethnicities, and between types of teeth [18–21]. Additional genetic analyses are required to replicate the initial published findings, to facilitate treatment of dental caries based on molecular or genetic information.

Given the high prevalence and specific characteristics of ECC, we performed a case-control study to clarify whether there were any associations between five VDR gene polymorphisms (rs1544410, rs731236, rs7975232, rs10735810, and rs11568820) and deciduous tooth caries, with the aim of exploring the combined impacts of VDR gene polymorphisms and environmental factors in the etiology of caries.

The article "Investigation of Interaction between Vitamin D Receptor Gene Polymorphisms and Environmental Factors in Early Childhood Caries in Chinese Children" was published in 2019. Journal: Biomed Res Int.

## 2. Materials and Methods

### 2.1. Study Subjects

This research was approved by the Ethics Committee of the Stomatological Hospital of Shandong University (Ethical committee number: R20180202). The study was performed under the guidelines of the World Medical Association Declaration of Helsinki. Informed consent was acquired from all children and their guardians. Chinese children (*n* = 549) aged 3–5 years were recruited from the same district of the city of Jinan for this study. The inclusion criteria were as follows: child aged 3–5 years old; Han ethnicity; mother lived in Jinan during the entire pregnancy and the child was raised in Jinan; mother had no pregnancy-related disease; and child did not have any systemic disease. The exclusion criteria were according to the published study performed by Antunes et al. [22]. Subjects were divided into three groups according to risk of caries and based on decayed, missing due to caries, or filled teeth (dmft) index value: high risk (dmft> 4), moderate risk (dmft = 1–4), and caries-free (dmft = 0).

### 2.2. Questionnaire

At baseline, guardians were asked to provide detailed information about their children's demographic characteristics (sex and birth weight), dietary habits (bottle fed or not, and the content and frequency of sucrose in the diet), and oral hygiene practices (brushing frequency, whether guardians helped with brushing, and whether toothpaste contained fluoride). Details of the educational level of guardians were also obtained using the questionnaire.

### 2.3. Dental Examination

Teeth that were decayed, missing due to caries, or filled were recorded according to the modified World Health Organization 1997 caries diagnostic criteria. At the beginning of the oral examination, possible food debris was removed using a piece of sterilized cotton, and the teeth surfaces were gently dried by air scavenging before recording the condition of the caries. In the caries group, white-spot lesions were also recorded, but not included for calculation of the dmft index. No radiographs were taken. Caries examination and diagnosis were performed by two dentists, and examination consistency was ensured by examining 20 children before the initiation of the study. The kappa value for agreement between the two examiners was 0.84.

### 2.4. Cariostat Test

Plaque samples were collected from primary maxillary and mandibular buccal surfaces using a sterile cotton swab before cleaning the teeth. The swab was scrubbed across the tooth surface three or four times with a wiping movement. Cotton swabs were placed into ampules containing 2.5 mL of Cariostat test medium and incubated at 37°C for 48 h. Cariostat scores were evaluated by referencing the sample against seven standard color tubes provided by the manufacturer.

The article "Investigation of Interaction between Vitamin D Receptor Gene Polymorphisms and Environmental Factors in Early Childhood Caries in Chinese Children" was published in 2019. Journal: Biomed Res Int.

### 2.5. DNA Collection

Sterile buccal swabs were used to obtain DNA by swabbing the buccal mucosa and stored at room temperature before transporting to the laboratory within 1 day. Genomic DNA was extracted using a TIANamp Swab DNA Kit (TIANGEN Biotech, Beijing, China), according to the manufacturer's instructions. The isolated DNA was stored at −20°C until use.

### 2.6. VDR Genotyping by TaqMan® Assay

DNA was screened for the rs7975232, rs1544410, rs731236, rs10735810, and rs11568820 polymorphisms in the VDR gene using TaqMan® assays on a Roche LC480 (Roche Diagnostics, Penzberg, Germany). Primers were designed using Primer Premier 5 (Premier Biosoft Inter, Palo Alto, USA) (Table 1) and synthesized by Shanghai Shenggong Co. (Shanghai, China). PCR reaction mixtures and conditions were designed according to the manufacturer's instructions (B639274 BBI, Shanghai Shenggong Co, Shanghai, China). Genotyping fidelity was verified using positive control subjects in each 384-well plate and re-running ≥5% of samples, which generated 100% concordant results. Genotype identification was performed using LightCycler480 Gene Scanning Software (Roche Diagnostics, Penzberg, Germany) and was blinded, with no information on the phenotypes of the subjects available to the individual conducting genotyping. Identified genotypes of rs10735810 were CC, CT, and TT; those of rs1544410 were AA, AG, and GG; those of rs731236 were TT, TC, and CC; those of rs7975232 were AA, AC, and CC; and those of rs11568820 were GG, AG, and AA.

### 2.7. Statistical Analysis

Data were analyzed using SPSS for Windows version 17.0 software (SPSS, Inc., Chicago, IL, USA). Hardy-Weinberg equilibrium in the three groups was assessed using SHEsis software (http://analysis.bio-x.cn/myAnalysis.php) [23, 24]. Differences in the proportions of sex, dietary habits, oral hygiene practices, Cariostat values, allele frequencies, genotype frequencies, and rates of allele carriage were compared among all groups using the Chi-square or Fisher's exact test. Associations of genes with behavioral factors were assessed by binary logistic regression. A *P* value <0.05 was considered significant. Odds ratios and 95% confidence intervals (CIs) were calculated. Power analysis was performed during design of the case-control study using PASS15 software and indicated that 304 cases and 245 controls could achieve a statistical power >0.8 in the present study.

The article "Investigation of Interaction between Vitamin D Receptor Gene Polymorphisms and Environmental Factors in Early Childhood Caries in Chinese Children" was published in 2019. Journal: Biomed Res Int.

## 3. Results

### 3.1. Demographic Characteristics of the Study Subjects

Study groups were a caries-free group (dmft = 0; *n* = 245; 108 boys and 137 girls), a moderate caries risk group (dmft = 1–4; *n* = 156; 85 boys and 71 girls), and a high caries risk group (dmft > 4; *n* = 148; 65 boys and 83 girls). Mean ages were 4.27 ± 0.792, 4.23 ± 0.794, and 4.31 ± 0.790 years in the caries-free, moderate caries risk, and high caries risk groups, respectively. The three groups exhibited no significant differences in age (*χ*^2^ = 5.019, *P*=0.285) or sex (*χ*^2^ = 4.912, *P*=0.086) (Table 2). Dmft indices in the caries groups ranged from 1 to 20, with mean indices of 2.390 ± 1.000 for the moderate caries risk group and 8.38 ± 1.391 for the high caries risk group.

### 3.2. Analysis of Environmental Risk Factors

Environmental risk factors for caries are summarized in Table 2. Feeding pattern within 6 months after birth, breastfeeding duration, sleeping with night milk or nipple, and dessert consumption before sleeping were correlated with the occurrence of caries in this population (*P* < 0.05) (Table 2).

### 3.3. Acidogenic Activity of Dental Bacteria

Acidogenic activity of dental bacteria was evaluated using the Cariostat test, and the resulting data are presented in Table 2. There was a significant difference among the three analyzed groups (*χ*^2^ = 56.198, *P* < 0.001). In the high caries risk group, most children (83.8%) had high activity of acidogenic bacteria, according to the Cariostat test (value ≥ 1.5, pH < 5.1), and only 4.7% of children had low activity levels (value = 0–0.5, pH > 5.7). Furthermore, 47.8% of caries-free children had high acidogenic activity, while 23.7% of caries-free children and 11.5% of high caries risk children had medium acidogenic bacteria activity (value = 1.0, pH = 5.2–5.6).

### 3.4. Genetic Analysis

Allele frequency, genotype distribution, and carriage rates are summarized in Table 3. All five single nucleotide polymorphisms (SNPs) were in the Hardy-Weinberg equilibrium (*P* > 0.091).

Significant differences were detected in the allele frequency, genotype distribution, and carriage rate of rs10735810 among the three experimental groups. As the severity of caries increased, C allele frequency was markedly higher, while that of the T allele was significantly lower (*χ*^2^ = 8.952, *P*=0.011). Furthermore, the frequency of the rs10735810 CC genotype was clearly higher in the high caries risk group than in controls and the moderate caries risk group (39.2%, 25.6%, and 30.6%, respectively; *P*=0.028). Increased frequency of the CT and CC genotypes of the rs10735810 VDR gene polymorphism was associated with high risk of dental caries relative to the two other groups (*χ*^2^ = 6.715, *P*=0.036). Moreover, the frequency of the rs10735810 C allele was significantly higher in the high caries risk group than in controls and the moderate caries risk group (64.2%, 53.2%, and 54.9%, respectively; *P*=0.011).

The article "Investigation of Interaction between Vitamin D Receptor Gene Polymorphisms and Environmental Factors in Early Childhood Caries in Chinese Children" was published in 2019. Journal: Biomed Res Int.

By contrast, no significant differences were detected among rs11568820, rs731236, rs1544410, and rs7975232 genotypes or allele frequencies in the three experimental groups (*P* > 0.05).

### 3.5. Multivariate Analysis

Oral behavioral factors and Cariostat values (*P* < 0.05; Table 2) were included as variables in regression analyses, along with all SNP genotypes, to evaluate the combined impacts of genetic and environmental factors on caries susceptibility (Table 4). The results showed that activity of acidogenic dental bacteria, frequent sleeping with night milk or nipple, and dessert consumption before sleeping were linked with an increased risk of deciduous tooth decay (acidogenic bacteria: OR = 3.881, 95% CI = 2.382–6.322, *P* < 0.001; night milk or nipple sleep: OR = 1.655, 95% CI = 1.025–2.673, *P*=0.032; and dessert consumption before sleeping: OR = 3.643, 95% CI = 1.119–11.864, *P*=0.032). By contrast, the VDR polymorphisms rs7975232, rs731236, rs1544410, rs11568820, and rs10735810 were not associated with deciduous tooth decay (rs7975232: OR = 1.050, 95% CI = 0.754–1.462, *P*=0.774; rs731236: OR = 1.842, 95% CI = 0.696–4.876, *P*=0.219; rs1544410: OR = 0.956, 95% CI = 0.342–2.677, *P*=0.932; rs11568820: OR = 0.886, 95% CI = 0.663–1.132, *P*=0.29; and rs10735810: OR = 1.167, 95% CI = 0.889–1.533, *P*=0.266).

## 4. Discussion

Based on data from previous studies, the development of dental caries is established as associated with various factors, including genetic and environmental influences [9, 11]. Although caries risk factors are well understood, studies have reported that not all individuals who appear to be at high risk actually develop caries, indicating variation in individual susceptibility [9, 10]. According to the Fourth Chinese National Epidemiological Survey, the Significant Caries Index (SiC) was much higher than the mean dmft for children aged 3–5 years [3], and a third of individuals with higher mean dmft indices were considered to be a population extremely susceptible to caries [25]. We hypothesized that individuals who had more caries lesions would be genetically susceptible to caries. The VDR gene, which is a candidate gene related to dental caries, mediates the biological function of the major metabolite, Vit D, which is associated with enamel development [13, 26]. Polymorphisms in human VDR lead to phenotypically diverse inherited malformations of the tooth enamel [16]. Given the role of VDR in enamel formation, we hypothesized a possible contribution of VDR gene polymorphisms to dental caries. We performed a case-control study to clarify the association between these polymorphisms and deciduous tooth caries and to explore the combined impacts of gene polymorphisms and environmental factors in the etiology of caries. In this study, the subjects were divided into three groups with high caries risk, with moderate caries risk, and without caries, according to dmft index values. Five VDR SNPs, rs1544410, rs731236, rs7975232, rs10735810, and rs11568820, were genotyped using TaqMan® assays in this study. Genetic screening of individuals with different dmft index values could be both important and valuable for caries prevention and diagnosis.

The article "Investigation of Interaction between Vitamin D Receptor Gene Polymorphisms and Environmental Factors in Early Childhood Caries in Chinese Children" was published in 2019. Journal: Biomed Res Int.

In this study, based on univariate analysis, we found that the VDR gene polymorphism rs10735810 may be associated with susceptibility to primary tooth caries in Chinese Han children. The frequency of the rs10735810 CC genotype was clearly higher in the high caries risk group than in controls and the moderate caries risk group (39.2%, 25.6%, and 30.6%, respectively; *P*=0.028). The high risk dental caries group was associated with increased frequencies of the CT and CC genotypes of rs10735810, relative to the other two experimental groups (*χ*^2^ = 6.715, *P*=0.036). This finding was similar to the results reported by Yu et al. in a Chinese 12-year-old adolescent population [17]. The rs10735810 SNP is located close to the 5′-UTR region of the VDR gene, within the DNA-binding domain [27–30]. This polymorphism changes the first potential start codon in the VDR gene from ATG to ACG, resulting in a VDR protein that is shorter by three amino acids and more efficient at transactivating Vit D target genes [31], which may account for the association of the rs10735810 C allele with susceptibility to dental caries. The present study also found that the frequency of the T allele was significantly reduced as the severity of caries increased (*χ*^2^ = 8.952, *P*=0.011), suggesting that the T allele of rs10735810 may be a protective factor against caries.

By contrast, we did not detect any associations of the VDR polymorphisms rs7975232, rs731236, rs1544410, or rs11568820 with deciduous tooth decay. Associations of these polymorphisms with susceptibility to dental caries vary greatly among different regions, ethnicities, and types of teeth. Kong et al. [19] reported that rs1544410 was associated with the risk of deciduous tooth caries in Chinese children aged 4–7 years; however, in our investigation we only found an association with rs10735810. We speculate that this difference may be attributable to geographical variations; the present study was performed in Shandong, northern China, while that of Kong et al. [19] was conducted in Guangzhou, southern China. The methodological approaches applied may also have contributed to the different results; our data were obtained using TaqMan methodology, which is considered more accurate than the PCR-restriction fragment length polymorphism technique used by Kong et al. [19]. The current study also found no association of the rs731236 VDR polymorphism with caries, similar to the findings of Izakovicova et al. [21], but inconsistent with those of Cogulu et al. [20], who reported that rs731236 genotype was a potential marker for susceptibility to dental caries in Turkish children. This difference may reflect geographic and ethnic variations among VDR polymorphisms. The rs10735810 and rs731236 variants were reported as associated with susceptibility to permanent dental caries in previous studies [17, 18]. Our findings, along with those of Kong et al. [19], indicate that the VDR polymorphisms rs10735810 or rs1544410 are associated with risk of deciduous tooth caries. Genetic factors may have different effects on caries formation in primary and permanent teeth. The rs7975232 polymorphism was not found to be associated with dental caries susceptibility in recent reports [17, 19, 20]. In the present study, we also investigated the association between rs11568820 polymorphisms and caries susceptibility, and our findings were in accordance with those of Cogulu et al. [20].

The article "Investigation of Interaction between Vitamin D Receptor Gene Polymorphisms and Environmental Factors in Early Childhood Caries in Chinese Children" was published in 2019. Journal: Biomed Res Int.

Furthermore, we investigated the combined impacts of gene polymorphisms and environmental factors on the etiology of caries. In univariate analysis, feeding pattern within 6 months after birth, breastfeeding duration, sleeping with night milk or nipple, dessert consumption before sleeping, and activity of acidogenic dental bacteria were correlated with the occurrence of caries in this population (*P* < 0.05). Significant environmental factors and genotype data from all five VDR SNPs were included as variables in regression analyses to evaluate the combined impacts of genetic and environmental factors. Our results showed that susceptibility to caries was increased by 264.3% (OR = 3.643, 95% CI = 1.119–11.864; *P*=0.032) in children who ate dessert before sleeping compared with those who did not. Similar results were found in the Chinese Fourth National Study conducted in 2016, in that children who had dessert before going to bed had a higher probability of developing caries [3]. Improper feeding habits are considered important factors contributing to caries development [8, 32]. Frequent sleeping with night milk or nipple increased caries susceptibility by 65.5% (OR = 1.655, 95% CI = 1.025–2.673; *P*=0.032). Furthermore, early cariogenic bacterial infection is an important predisposing factor for ECC [33]. The Cariostat test was used to measure the acidogenic activity of bacteria isolated from the teeth of subjects in this study, which can indicate levels of infection with mutans streptococci and lactobacilli in plaque [34]. Subjects with Cariostat values of 1.5–3.0 showed significantly higher caries risk than those with values of 0–0.5 (OR = 3.881, 95% CI = 2.382–6.322; *P* < 0.001), increasing caries incidence by 288.1%.

The article "Investigation of Interaction between Vitamin D Receptor Gene Polymorphisms and Environmental Factors in Early Childhood Caries in Chinese Children" was published in 2019. Journal: Biomed Res Int.

Multivariate analysis indicated that none of the VDR polymorphisms tested were associated with deciduous tooth decay. Based on the results of this study, the VDR gene variants rs7975232, rs10735810, rs1544410, rs11568820, and rs731236 are not suitable markers for identification of Chinese children with increased dental caries risk, when combined with environmental caries risk factors. However, caries is a multifactorial disease, which is affected by many environmental factors. Vit D is associated with enamel development [13, 26], and the synthesis of vitamin D is affected by sunlight exposure time. The limitation of this study did not mention the relationship between the sunlight exposure time and caries risk. Future studies in different populations and regions are needed to replicate these initial findings and to better assess the risk of caries in deciduous teeth.

## 5. Conclusion

In conclusion, we investigated both oral behavioral habits and the difference in distribution of VDR polymorphic loci in children with different caries risk. Improper feeding habits, with night milk feeding or nipple, dessert consumption before sleeping, and high activity of acidogenic dental plaque bacteria were associated with increased caries risk. However, none of the VDR gene variants were suitable markers for identification of Chinese Han children with increased primary tooth caries risk. Future studies in different populations and regions are needed to replicate these initial findings and to better assess the risk of caries in deciduous teeth.

## Figures and Tables

**Table 1:** Primers and MGB probes for VDR gene polymorphisms.

Candidate gene	Primer	Fragment length (bp)	MGB probe	Probe direction
FokI (rs10735810)	5′-CTGGCACTGACTCTGGCTCT-3′	88 bp	5′-FAM-TTGCCTCC[A]TCCCT-3′MGB	Reverse
	5′-GGGTCAGGCAGGGAAGTG-3′		5′-VIC-TTGCCTCC[G]TCCCT-3′MGB	

TaqI (rs731236)	5′-TTCTCTATCCCCGTGCCC-3′	97bP	5′-FAM-CGCTGAT[C]GAGGC-3′MGB	Forward
	5′- TGTACGTCTGCAGTGTGTTGG- 3′		5′-VIC-CGCTGAT[T]GAGGCC-3′MGB	

Bsm I (rs1544410)	5′-GGATTCTGAGGAACTAGATAAGCA 3′	91bP	5′-FAM-CCTGC[A]CATTCC-3′MGB	Forward
	5′-CCAGTTCACGCAAGAGCAG-3′		5′-VIC-CCTGC[G]CATTCC-3′MGB	

ApaI (rs7975232)	5′-GGCACGGGGATAGAGAAGA-3′	96 bp	5′-FAM-CTGGGC[A]CCTCAC-3′MGB	Forward
	5′-GCTGCCGTTGAGTGTCTGT-3′		5′-VIC-CTGGGC[C]CCTCAC-3′MGB	

CdX-2 (rs11568820)	5′-AGAACATCTTTTGTATCAGGAACTT-3′	98 bp	5′-FAM-CTAGGTCACA[A]TAAAA-3′MGB	Forward
	5′-TTCAAAATTTTAACTGCAACCC-3′		5′-VIC-CTAGGTCACA[G]TAAAA-3′MGB	

The article "Investigation of Interaction between Vitamin D Receptor Gene Polymorphisms and Environmental Factors in Early Childhood Caries in Chinese Children" was published in 2019. Journal: Biomed Res Int.

**Table 2:** Demographic characteristics and environmental risk factors for caries in the studied population.

Variables	Caries-free group (*n* = 245)	Moderate caries risk group (*n* = 156)	High caries risk group (*n* = 148)	*χ* ^2^	*P*
Age				5.019	0.285
3 years	70 (28.6)	35 (22.4)	30 (20.3)		
4 years	71 (29.0)	50 (32.1)	42 (28.4)		
5 years	104 (42.4)	71 (45.5)	76 (51.4)		

Gender (male/female)	108/137 (44.1/55.9)	85/71 (54.5/45.5)	65/83 (43.9/56.1)	4.912	0.086

Birth weight				—^*∗*^	0.452
<2.5 kg/≥2.5 kg	5/235 (2.1/97.9)	3/148 (2.0/98.0)	6/14 (4.1/95.9)		
Missing	5	5	1		

Time of first tooth eruption				9.129	0.058
≤6 mos	120 (56.3)	100 (69.0)	85 (62.5)		
6–8 mos	69 (32.4)	29 (20.0)	31 (22.8)		
≥9 mos	24 (11.3)	16 (11.0)	20 (14.7)		
Missing	32	11	12		

Father's education level				1.219	0.875
Elementary	12 (4.9)	7 (4.5)	4 (2.7)		
High school	24 (9.8)	16 (10.3)	16 (10.8)		
College and higher	209 (85.3)	133 (85.3)	128 (86.5)		

Mother's education level				5.142	0.273
Elementary	16 (6.5)	6 (3.8)	3 (2.0)		
High school	27 (11.0)	19 (12.2)	21 (14.2)		
College and higher	202 (82.4)	131 (84.0)	124 (83.8)		

Feeding pattern before 6 mos old (%)				18.614	0.017
Exclusively breastfed	76 (31.0)	56 (35.9)	69 (46.6)		
Predominantly breastfed	68 (27.8)	36 (23.1)	44 (29.7)		
Exclusively formula fed	22 (9.0)	11 (7.1)	4 (2.7)		
Predominantly formula fed	22 (9.0)	13 (8.3)	7 (4.7)		
Mixed fed (50/50)	57 (23.3)	40 (25.6)	24 (16.2)		

Breast feeding duration				22.795	0.001
≤6 mos	70 (28.9)	38 (24.5)	17 (11.5)		
6–12 mos	53 (21.9)	49 (31.6)	37 (25.0)		
12–18 mos	74 (30.6)	38 (24.5)	58 (39.2)		
≥18 mos	45 (18.6)	30 (19.4)	36 (24.3)		
Missing	3	1			

Mouth-to-mouth or chewing to feed				—^*∗*^	0.882
Often	2 (0.8)	1 (0.6)	2 (1.4)		
Occasionally	43 (17.6)	32 (20.5)	26 (17.6)		
Never	200 (81.6)	123 (78.8)	120 (81.1)		

Night milk or nipple sleep				9.661	0.047
Often	47 (19.2)	44 (28.2)	46 (31.1)		
Occasionally	78 (31.8)	52 (33.3)	43 (29.1)		
Never	120 (49.0)	60 (38.5)	59 (39.9)		

Dessert consumption before sleeping				21.405	<.001
Often	5 (2.0)	6 (3.8)	9 (6.1)		
Occasionally	113 (46.1)	84 (53.8)	96 (64.9)		
Never	127 (51.8)	66 (42.3)	43 (29.1)		

Milk consumption before sleeping				4.237	0.375
Often	80 (32.7)	57 (36.5)	54 (36.5)		
Occasionally	107 (43.7)	70 (44.9)	71 (48.0)		
Never	58 (23.7)	29 (18.6)	23 (15.5)		

Dessert or candy intake frequency				7.550	0.110
Less often than daily	208 (84.9)	119 (76.3)	111 (75.0)		
Once a day	26 (10.6)	24 (15.4)	24 (16.2)		
Twice a day or more	11 (4.5)	13 (8.3)	13 (8.8)		

Sweet or acidic drinks intake frequency				—^*∗*^	0.992
Less often than daily	237 (96.7)	150 (96.2)	144 (97.3)		
Once a day	5 (2.0)	4 (2.6)	3 (2.0)		
Twice a day or more	3 (1.2)	2 (1.3)	1 (0.7)		

Milk with sugar intake frequency				2.062	0.724
Less often than daily	192 (78.4)	127 (81.4)	123 (83.1)		
Once a day	46 (18.8)	24 (15.4)	20 (13.5)		
Twice a day or more	7 (2.9)	5 (3.2)	5 (3.4)		

Toothbrushing (yes/no)	191/54 (78.0/22.0)	118/38 (75.6/24.4)	126/22 (85.1/14.9)	4.598	0.100
Age when toothbrushing started				5.565	0.062
≤12 mos/>12 mos	72/173 (29.4/0.6)	34/122 (21.8/78.2)	29/118 (19.7/80.3)		

Tooth brushing frequency			6.169	0.187	
Twice per day	47 (19.2)	26 (16.7)	37 (25.0)		
Once per day	122 (49.8)	88 (56.4)	78 (52.7)		
Occasionally or never	76 (31.0)	42 (26.9)	33 (22.3)		

Adult-assisted toothbrushing				4.295	0.637
Every day	52 (21.3)	32 (20.5)	35 (24.0)		
Often	88 (36.1)	59 (37.8)	54 (37.0)		
Occasionally	76 (31.1)	49 (31.4)	49 (33.6)		
Never	28 (11.5)	16 (10.3)	8 (5.5)		
Missing	1		2		

Brushing with toothpaste				3.744	0.154
Yes/no	229/14 (94.2/5.8)	146/10 (93.6/6.4)	145/3 (98.0/2.0)		
Missing	2				

Fluoride toothpaste or not				2.157	0.707
Yes	55 (22.6)	33 (21.2)	32 (21.6)		
No	124 (51.0)	90 (57.7)	77 (52.0)		
Do not know^&^ amp	64 (26.3)	33 (21.2)	39 (26.4)		
Missing	2				

Cariostat value				56.198	<.001
0–0.5	70 (28.6)	26 (16.7)	7 (4.7)		
1.0	58 (23.7)	25 (16.0)	17 (11.5)		
1.5–3.0	117 (47.8)	105 (67.3)	124 (83.8)		

^&^Do not know: do not know if the toothpaste used contains fluoride. ^*∗*^When cells had expected count <5, Fisher's exact test was used.

The article "Investigation of Interaction between Vitamin D Receptor Gene Polymorphisms and Environmental Factors in Early Childhood Caries in Chinese Children" was published in 2019. Journal: Biomed Res Int.

**Table 3:** Allele and genotype frequencies of five VDR gene polymorphisms of the participants.

		Caries-free group (*n* = 245)	Moderate caries risk group (*n* = 156)	High caries risk group (*n* = 148)	*χ* ^2^	*P*
CdX-2	A	198 (40.4)	138 (44.2)	125 (42.5)	1.177	0.555
	G	292 (59.6)	174 (55.8)	169 (57.5)		
	AA/AG/GG	37/124/84 (15.1/50.6/34.3)	28/82/46 (17.9/52.6/29.5)	31/63/53 (21.1/42.9/36.1)^#^	4.648	0.325
	Carriage of allele A	161 (65.7)	110 (70.5)	94 (63.9)	1.626	0.444

Fok I	C	269 (54.9)	166 (53.2)	190 (64.2)	8.952	0.011
	T	221 (45.1)	146 (46.8)	106 (35.8)		
	CC/CT/TT	75/119/51 (30.6/48.6/20.8)	40/86/30 (25.6/55.1/19.2)	58/74/16 (39.2/50.0/10.8)	10.899	0.028
	Carriage of allele C	194 (79.2)	126 (80.8)	132 (89.2)	6.715	0.035
	Carriage of allele T	170 (69.4)	90 (60.8)	116 (74.4)	6.625	0.036

Taq I	C	39 (8.0)	14 (4.5)	17 (5.7)	4.191	0.123
	T	449 (92.0)	298 (95.5)	279 (94.3)		
	CC/TT/TC	1/37/206 (0.4/15.2/84.4)#	0/14/142 (0.0/9.0/91.0)	1/15/132 (0.7/10.1/89.2)	—^*∗*^	0.197
	Carriage of allele C	38 (15.6)	14 (9.0)	16 (10.8)	4.289	0.117

Bsm I	A	33 (6.7)	12 (3.8)	16 (5.4)	3.049	0.218
	G	457 (93.3)	300 (96.2)	280 (94.6)		
	AA/AG/GG	1/31/213 (0.4/12.7/86.9)	0/12/144 (0.0/7.7/92.3)	0/16/132 (0.0/10.8/89.2)	—^*∗*^	0.401
	Carriage of allele A	32 (13.1)	12 (7.7)	16 (10.8)	2.825	0.244

Apa I	A	142 (29.1)	78 (25.2)	85 (28.7)	1.603	0.449
	C	346 (70.9)	232 (74.8)	211 (71.3)		
	AA/AC/CC	21/100/123 (8.6/41.0/50.4)#	9/60/86 (5.8/38.7/55.5)^#^	8/69/71 (5.4/46.6/48.0)	3.864	0.425
	Carriage of allele A	121 (49.6)	69 (44.5)	77 (52.0)	1.816	0.403

^*∗*^When cells had expected count <5, Fisher's exact test was used. ^#^Using MGB-TaqMan® genotyping method, 1 subject in the high caries risk group had negative result of Cdx-2. 1 subject in the caries free group had negative result of Taq I. 1 subject in the caries-free group and 1 subject in the moderate caries risk group had negative result of Apa I.

**Table 4:** Multivariate analysis of genotypes and behavioral factors in the subjects.

Covariables	*β*	*P*	OR	95% CI for OR	
				Lower	Upper
Apa I genotype	0.049	0.774	1.050	0.754	1.462
Bsm I genotype	−0.045	0.932	0.956	0.342	2.677
CdX-2 genotype	−0.143	0.293	0.866	0.663	1.132
Fok I genotype	0.155	0.266	1.167	0.889	1.533
Taq I genotype	0.611	0.219	1.842	0.696	4.876
Feeding pattern before 6 mos old (%)	−0.187	0.052	0.830	0.687	1.002
Breast feeding duration	−0.016	0.886	0.984	0.792	1.223
Night milk or nipple sleep		0.115			
Often	0.504	0.039	1.655	1.025	2.673
Occasionally	0.124	0.577	1.131	0.733	1.746
Never	Reference				
Dessert consumption before sleeping	0.002				
Often	1.293	0.032	3.643	1.119	11.864
Occasionally	0.612	0.001	1.845	1.266	2.687
Never	Reference				
Cariostat value		<0.001			
1.5–3.0	1.356	<0.001	3.881	2.382	6.322
1.0	0.341	0.265	1.406	0.772	2.559
0–0.5	Reference				
Constant	−2.515	0.015	0.081		

## Data Availability

The data used to support the findings of this study are available from the corresponding author upon request.
